# RNAi-mediated *TCF-3* gene silencing inhibits proliferation of Eca-109 esophageal cancer cells by inducing apoptosis

**DOI:** 10.1042/BSR20170799

**Published:** 2017-11-09

**Authors:** Jie Ma, Xian-Bin Wang, Rui Li, Shu-Hong Xuan, Fang Wang, Xin-Hua Li, Zhi-Ping Zhang, Lu Tan, Lian Li

**Affiliations:** 1 Department of Oncology, Jining No. 1 People’s Hospital, Jining 272011, P.R. China; 2 Department of Breast and Thyroid Surgery, Jining No. 1 People’s Hospital, Jining 272011, P.R. China; 3 Department of Neurology, Jining No. 1 People’s Hospital, Jining 272011, P.R. China; 4 Department of Internal Medicine, Jining No. 1 People’s Hospital, Jining 272011, P.R. China; 5 Department of Oncology, The Second Hospital of Shandong University, Jinan 250033, P.R. China

**Keywords:** Cell cycle, Esophageal cancer, Eca-109 cell, Proliferation, SiRNA, Transcription factor 3 gene

## Abstract

Esophageal cancer (EC) remains an important health problem in China. In the present study, through the use of siRNA, specific gene knockdown of transcription factor 3 gene (*TCF-3*) was achieved *in vitro* and the effect of *TCF-3* gene on human EC Eca-109 cell proliferation and apoptosis. Eca-109 cells were treated using negative control (NC) of siRNA against TCF-3 (siTCF-3) and siTCF-3 group. Colony formation assay was used to detect the colony formation ability in Eca-109 cells. MTT assay was used to measure the cell growth and viability, whereas BrDU assay was used to evaluate cell proliferation, and flow cytometry (FCM) to assess cell apoptosis. Reverse-transcription quantitative PCR (RT-qPCR) was applied to measure *TCF-3* gene expression. Protein expressions of TCF-3, apoptosis-related proteins, Bcl-2, Bax, and caspase-3 were determined using Western blotting. Transfection of siTCF-3 successfully down-regulated *TCF-3* gene expression. In addition, siTCF-3, reduced Eca-109 cell viability and proliferation, in a time-dependent manner, and inhibited progression of cell cycle from G_0_/G_1_ to S-stage. When treated with siTCF-3, the Eca-109 cells exhibited increased apoptosis, with up-regulated cleaved caspase and Bax expressions, whereas Bcl-2 expression was down-regulated. The present study shows that *TCF-3* gene silencing inhibits Eca-109 cell growth and proliferation, suppresses cell cycle progression, and promotes apoptosis, which might serve as a new objective for EC treatment.

## Introduction

Esophageal cancer (EC), mostly occurs as esophageal squamous cell carcinoma, which is the eighth most common type of cancer all over the world with 482300 new cases every year. It is also the leading cause of cancer-related deaths with 406800 cases recorded in 2008 all over the world [1]. It is reported that squamous cell carcinoma is the most common histological type of EC in the world, which occupies a higher incidence in developing countries [2]. Eastern Asia is one of the areas with the highest incidence rate, and men are three to four times more likely to develop EC than women. [3]. Traditional therapies such as surgery, chemotherapy, and radiotherapy have been regarded as effective treatments for EC, however, the serious side effects and long-term survival showed that these therapies had poor prognosis after surgery [4,5]. Nowadays, regulatory factors such as miRNAs, genes, and signaling pathways have provoked wide concern in treating cancer as it is safer than traditional therapies due to fewer side effects [6-8]. Abnormal gene expressions are associated with the advanced stages of EC, and gene silencing could inhibit the growth and development of EC tumors [9,10]. Accordingly, various types of gene silencing might have a potential in suppressing EC [11,12].

Transcription factor 3 (TCF-3) is a conserved transcription factor that functions as a transcriptional repressor by interacting with β-catenin [13]. TCF-3 is mostly related to the regulation of embryonic and epidermal stem cell identity, as well as in the initiation and further growth of tumors [14]. TCF-3 also plays a major role in apoptosis or proliferation of many cells [15,16]. TCF-3 protein acts as a DNA-binding transcriptional regulator along with Wnt signaling pathway. When Wnt-stabilized β-catenin accumulates in cells, it enhances the transcription of downstream targets [17]. TCF-3 acts on its domain that interacted with β-catenin to inhibit epidermal terminal differentiation, in which TCF-3 is generally shut off, and enhances multipotent stem cells (bulge) [18]. And, as a platform, TCF-3 has been revealed to primarily suppress expression of Wnt target genes by exchanging corepressors with co-activators [19]. It is possible that TCF-3 might have some effect on EC, therefore, in the present study, we transfected Eca-109 cells with siRNA and then studied the correlation between *TCF-3* gene silencing and the proliferation and apoptosis of Eca-109 cells.

## Materials and methods

### Cell culture

The EC cell line Eca-109, purchased from Cell Bank of the Shanghai Institutes for Biological Sciences, Chinese Academy of Sciences, was cultured in 1640 medium (Gibco BRL Co., Ltd., Gaithersburg, MD, U.S.A.) with 1% double antibody (100 U/l penicillin and 100 mg/l streptomycin, Gibco BRL Co., Ltd., Gaithersburg, MD, U.S.A.) containing 10% FBS (Tianhang Biological Technologies Inc., Zhejiang, China), later cells were cultured at 37°C with 5% CO_2_. Reading of the cells was taken once every 2–3 days, and then cells in the logarithmic growth phase were collected for the following experiment.

### Cell treatment

Eca-109 cells in the logarithmic growth phase were inoculated into six-well plates for 24 h, and then cultured in the medium without antibiotic. When the cell density reached 40–60%, cells were cultured in Opti-MEM medium without serum. Cells were transfected after reaching 70% convergence, and the compound of transfection reagent and siRNA (200 μl) were arranged in accordance with the instruction of Lipofectamine 2000 Transfection Kit (Invitrogen Inc., Carlsbad, CA, U.S.A.), which was then added into the medium. A negative sequence without interference was transfected as a control. After transfection, the cells were cultured at 37°C with 5% CO_2_, followed by the replacement of the medium with 1.5 ml of normal medium containing serum after 6-h culture. The cells were divided into control group, negative control group (NC group, with non-specific siRNA-NC), and siRNA against TCF-3 (siTCF-3)-1 group, siTCF-3-2 group, and siTCF-3-3 group (with *TCF-3* gene silenced by RNAi 1, RNAi 2, RNAi 3). All siRNA sequences were synthesized by Shanghai GenePharma Co., Ltd. Shanghai, China. Sequences of siTCF-3-1, siTCF-3-2, and siTCF-3-3 are shown in Table 1. Forty-eight hours after the cell treatment, the mRNA level of TCF-3 in Eca-109 cells was determined by reverse-transcription quantitative PCR (RT-qPCR) to screen the best siTCF-3 for later experiments (Table 1).

**Table 1:** The sequences of three siTCF-3

Gene	Sequence (5′–3′)
siTCF3-1	Forward: CACUCCAGCAAUAAUUUCUUU
	Reverse: AGAAAUUAUUGCUGGAGUGUU
siTCF3-2	Forward: CUGGACUUCAGCAUGAUGUUU
	Backward: ACAUCAUGCUAAAGUCCAGUU
siTCF3-NC	Forward: UUCUCCGAACGUGUCACGUUU
	Backward: ACGUGACACGUUCGGAGAAUU

### Colony formation assay

The Eca-109 cells in the logarithmic growth phase were digested into cell suspension after being washed by PBS twice. After counting, the cells were diluted to achieve a suitable density, and then a specific number of cells were inoculated in a culture dish with a diameter of 60 mm in accordance with different exposure doses. Three duplicated wells were set for each exposure dose. Then, the cells were treated in different groups and were cultured in an incubator for 10–14 days. On the 14th day, cells were suspended in methanol for 30 min, and dyed using 0.1% Crystal Violet for 15 min. The colony forming cells were photographed via a low power microscope, and the total number was counted, then the average and formation rates of colony forming cells were measured.

### MTT assay

The Eca-109 cells in the logarithmic growth phase were suspended again in the cell growth medium. Cell density was adjusted to 10^4^ cells/ml, and then the cells were put in a 96-well plate, with 100 μl in each well. The medium was abandoned and different siRNAs were added 24 h later after cell adhesion, with three duplicated well sets. After 6 h, cells were cultured in a normal medium, and after 24, 48, and 72 h of culture, respectively, each well was added with 10 μl MTT (Sigma–Aldrich Chemical Company, St. Louis, MO, U.S.A.) (away from light) for incubation for another 4 h. The culture liquid in the 96-well plate was then absorbed carefully, and then, 10 μl of DMSO (Sigma–Aldrich Chemical Company, St. Louis, MO, U.S.A.) was added in each well (in the dark). Shaken and dissolved on a plate agitator for 15 min, the cells were detected using a microplate reader. The optical density (OD) at 570 nm was noted and the growth activity of Eca-109 cell (the effect of *TCF-3* gene silencing on the growth of Eca-109 cell) was measured. At the same time, the changes in the morphology of the cells before culturing and after *TCF-3* gene silencing were observed via an inverted microscope.

### BrDU assay

The Eca-109 cells in the logarithmic growth phase were resuspended in the cell growth medium. Cell density was adjusted to 1.0 × 10^4^ cells/ml, and then cells were seeded in 24-well plates with cover glass, 3 ml in each well. The medium was abandoned and different siRNAs were added 24 h later after incubation, with three duplicated well sets. Twenty-four hours after incubation, the cover glass was washed thrice with PBS in 3 min. Then, immersed in 4% formaldehydum polymerisatum and incubated at room temperature for 15 min, the cover glass was washed again thrice with PBS in 3 min. After osmotic treatment with 0.05% Triton X-100 (ST795, Beyotime Biotechnology Co., Ltd., Shanghai, China) for 20 min, the samples were incubated with 2 mol/l HCL at room temperature for 1 h, and washed with PBS thrice in 5 min. Next, the samples were immersed in 0.1 M Na_2_B_4_O_7_ (equal to 2 mol/l HCL) at room temperature for 15 min, and washed with PBS thrice in 10 min. Then, PBS was blotted by absorbent paper and normal goat serum was added drop by drop. Sufficient amount of well-diluted primary antibody of BrDU was added into each glass (1:50, ab187275, Abcam Inc., Cambridge, MA, U.S.A.) and incubated at 4°C in a wet box overnight. The glass was washed with PBS containing Tween (PBST) thrice in 3 min. Then, the surplus liquid was blotted by absorbent paper. Subsequently, the samples were added with diluted goat anti-rat IgG-CY3 (1:100, BA1031, Wuhan Boster Biological Technology Ltd., Wuhan, Hubei, China), placed in a wet box, and incubated at 20–37°C for 1 h. The glass was washed again with PBST thrice in 3 min, and DAPI (C1002, Beyotime Biotechnology Co., Ltd., Shanghai, China) was added to incubate in the dark for 5 min, the nuclei of specimens were stained, and washed with PBST four times in 5 min to remove the surplus DAPI. Then, the absorbent paper was used to blot the liquid on the glass, and affixed in the sealing agents containing anti-fluorescence quenching agents (0100-01, SouthernBiotech Inc., Birmingham, U.S.A.). The images were observed under the fluorescence microscope (Olympus BX71, Tokyo, Japan) (200×).

### Propidium iodide staining and flow cytometry

The Eca-109 cells in the logarithmic growth phase were put in a six-well plate with a cell density of 1.2 × 10^5^ cells/ml, with 2 ml for each well. Twenty-four hours later, the cells were transfected with different standards after reaching 70–80% confluence, and the culture liquid was changed after being transfected for 6 h. Subsequently, the cells were collected by trypsinization without EDTA and centrifuged at 2500 rpm for 5 min. The cells were then washed with PBS twice, then collected, and immersed in 3 ml 70% ethanol and preserved overnight at 4°C. The next day, the cells were stained using propidium iodide (PI) after centrifugation and supernatants were removed. After staining, the cells were filtered, and the ratio of cells in G_0_/G_1_, S, and G_2_/M-phases was measured using flow cytometry (FCM) (Becton Dickinson and Company, NJ, U.S.A.).

### Annexin-V/PI double staining and FCM

The cells were collected by trypsinization without EDTA. After centrifugation at 2500 rpm for 5 min, the cells were washed with cold-PBS twice. Then the certain number of cells (1 × 10^6^) were transferred into Eppendorf (EP) tubes. Each tube was added with 500 μl binding buffer, 5 μl PI (Nanjing KeyGen Biotech Co. Ltd., Nanjing, China), and 5 μl Annexin-V (Nanjing KeyGen Biotech Co. Ltd., Nanjing, China). Then the cells were incubated in the dark for 10–15 min after the addition of dye, and 400-mesh cell strainer was used to filter the cell suspension. Cells were then put on ice and detected by FCM (Becton Dickinson and Company, NJ, U.S.A.) within 30 min.

### RT-qPCR

Eca-109 cells of each group were collected and the total RNA present in the cell was extracted using TRIzol reagent to measure the concentration of RNA. RNA was used to generate cDNA using reverse transcription (a total system of 10 μl) according to the instructions on Reverse Transcription Kit (Takara Biotechnology Ltd., Dalian, China). The cDNA was diluted with 65 μl diethyl phosphorocyanidate (DEPC) and then mixed uniformly. The PCR reaction included 5 μl SsoFast EvaGreen Supermix (2×), 0.5 μl forward primers (10 μM), 0.5 μl reverse primers (10 μM), and 4 μl cDNA. The conditions required were predenaturation at 95°C for 1 min, then denaturation at 95°C for 30 s, and annealing at 58°C for 5 s, followed by 30 cycles and extension at 65–95°C for 5 s. The primers were synthetized by Beijing Genomics Institute (Shenzhen, China) (Table 2).

**Table 2:** Primer sequences for quantitative real-time PCR

Gene	Primer sequence (5′–3′)
*TCF-3*	Forward: TGAGAAGCCTTGTGATAGCC
	Reverse: GAGACAGCCTGCATAGAACC
*GAPDH*	Forward: GGTGAAGGTCGGAGTCAACG
	Reverse: CAAAGTTGTCATGGATGHAC

Abbreviation: GAPDH, glyceraldehyde-3-phosphate dehydrogenase.

### Western blotting

Cells were collected by trypinization, and then added with an appropriate amount of cell lysis (SDS:PMSF) after cells were centrifuged and washed with PBS twice. After cell lysis for 30 min at 12000 rpm on ice and centrifugation at 4°C for 20 min, the cell lysate was adequately centrifuged and then the supernatant, which consisted of the total protein in the cells, was collected and transferred into EP tubes. The protein concentration in each group was determined using BCA protein assay kit and was adjusted to the same level. Protein extraction was quantitated, then added with 5× SDS loading buffer, and denatured at 95°C for 5 min, followed by SDS/PAGE. After electrophoresis, then transferred on to membrane, 5% skimmed milk was added to the sample and reserved hermetically at 4°C overnight. After membranes were cleaned using TBS with Tween 20 (TBST), extracted protein continued to be added with primary antibodies TCF-3 (#2883, Cell Signaling Technology (CST), Beverly, MA, U.S.A.), Bcl-2 (#2870, CST, Beverly, MA, U.S.A.), Bax (#5023, CST, Beverly, MA, U.S.A.), cleaved-caspase-3 (#9665, CST, Beverly, MA, U.S.A.), and glyceraldehyde-3-phosphate dehydrogenase (GAPDH, as an internal reference) for incubation overnight. After membranes were cleaned using TBST, the sample was added with the secondary antibody horseradish peroxidase (HRP) and incubated at 37°C for 1 h. The sample was eventually developed with HRP ECL after membranes were cleaned again using TBST. Then, a photographic film was produced, which was washed by water, and then scanned and recorded after drying.

### Statistical analysis

Data were analyzed using the Statistical Package for the Social Sciences (SPSS) version 21.0 (SPSS Inc., Chicago, IL, U.S.A.). Each experiment was repeated at least three times and the average value and S.D. were calculated. Comparison between the two groups was studied using *t* test, whereas multiple groups were compared using one-way ANOVA. The level of significant difference was set as *P*<0.05 and the level of immense significant difference was set as *P*<0.01.

## Results

### siTCF-3-2 exhibited better inhibitory effect on TCF-3 expression than siTCF-3-1

Forty-eight hours after the liposome was transfected with Eca-109 cells, RT-qPCR was used to detect *TCF-3* mRNA level, which revealed that compared with the control and siRNA/control (si-NC) groups, the mRNA levels of TCF-3 in the siTCF-1, and siTCF-2 groups remarkably decreased, (all *P*<0.01), but there was no significant difference in the mRNA level between control and NC groups (*P*>0.01) (Figure 1A). Figure 1B showed that by taking the control group as a reference, the inhibition rate of siTCF-3-2 group was significantly higher than that of the siTCF-3-1 group (all *P*<0.01). Therefore, siTCF-3 group (named as siTCF-3 group) was chosen for further experiments.

**Figure 1:** mRNA relative expression of TCF-3 after transfection (**A**) The mRNA relative expression of TCF-3 in Eca-109 cells after transfection; (**B**) the silencing efficiency of siTCF-3-1 and siTCF-3-2 in Eca-109 cells; **, *P*<0.01 compared with the control group; ^#^, *P*<0.01 compared with the siTCF-3-1 group.

### Down-regulation of TCF-3 affects Eca-109 cell morphology

The morphological changes in the cells before and after transfection with siTCF-3 were observed using an inverted microscope. The results showed that after transfection, the morphology and density of cells significantly changed. In the control and NC groups, cells were in normal shape, with clear outlines and bright bodies. Compared with the control and NC groups, Eca-109 cells in the siTCF-3 group were irregular with cell membrane crinkled and broken, cells dropped from the bottom of the plate and the cell density decreased due to many dead cells (Figure 2).

**Figure 2:** The morphology changes of Eca-109 cells amongst control, NC, and siTCF-3 groups

### Down-regulation of TCF-3 inhibits Eca-109 cell viability and colony formation

The result of MTT assay showed that *TCF-3* gene silencing could inhibit the proliferation of Eca-109 cells, and the rate of inhibition eventually improved with time and was the highest at 72 h. No such significant difference was found between the control group and the NC group (*P*=0.68, *P*=0.73) (Figure 3). The result of colony formation assay proved that the colony formation ability of Eca-109 cells in each group was distinctly different. Compared with the control group, the colony formation ability of Eca-109 cells in the NC group showed no difference (*P*>0.05), while that in the siTCF-3 group significantly reduced (*P*<0.05) (Figure 4).

**Figure 3:** Eca-109 cell viability amongst control, NC, and siTCF-3 groups **, *P*<0.01 compared with the control group.

**Figure 4:** Eca-109 cell colony formation abilities amongst control, NC, and siTCF-3 groups (**A**) Colony morphology; (**B**) efficiency of colony formation; **, *P*<0.01 compared with the control group.

### Down-regulation of TCF-3 inhibits Eca-109 cell proliferation

The BrDU assay demonstrated that *TCF-3* gene silencing inhibited the Eca-109 cells proliferation (Figure 5). There was no significant difference in the number of BrDU-positive cells between the control and the NC groups (*P*>0.01), but the number of BrDU-positive cells in the siTCF-3 group was significantly lower than that in the control group and the NC group (*P*<0.01).

**Figure 5:** Proliferation of Eca-109 cells amongst control, NC, and siTCF-3 groups (**A**) BrDU-stained cells under the fluorescence micrograph; (**B**) the number of BrDU-stained cells; **, *P*<0.01 compared with the control group.

### Down-regulation of TCF-3 suppresses Eca-109 cell cycle progression

The ratio of Eca-109 cells in G_0_/G_1_-phase in the siTCF-3 group was higher than that in the control and NC groups (*P*=0.01, *P*=0.01). The ratio of cells in the siTCF-3 group in S-phase was lower than that in the control and NC groups (*P*=0.01, *P*<0.01). No significant difference was found between control group and NC group (*P*=0.68, *P*=0.73). Eca-109 cells in G_2_-phase in each group showed no statistical difference (*P*=0.12, *P*=0.13). The results showed that *TCF-3* gene silencing could arrest Eca-109 cells in G_0_/G_1_-phase (Figure 6).

**Figure 6:** The cell cycle of Eca-109 cells amongst control, NC, and siTCF-3 groups (**A**) The number of Eca-109 cells in G_0_/G_1_, S, and G_2_-phases; (**B**) Ratios of Eca-109 cells in G_0_/G_1_, S, and G_2_-phases; **, *P*<0.01 compared with the control group.

### Down-regulation of TCF-3 facilitates Eca-109 cell apoptosis

Compared with the control group, no significant difference in cell apoptosis was shown in the NC group, while cell apoptosis was induced in the siTCF-3 group and the apoptosis rate increased significantly (*P*<0.01). In comparison with the control group, the apoptosis-related proteins revealed no significant difference in the NC group, while in the siTCF-3 group, the cell apoptosis-related signaling pathway was activated, thus the apoptosis-related protein caspase-3 was cleaved, and the cleaved-caspase-3 distinctly improved, expression of anti-apoptotic protein Bcl-2 decreased, and the expression of proapoptotic protein Bax increased. These results proved that *TCF-3* gene silencing could promote apoptosis of Eca-109 cells (*P*<0.01) (Figure 7).

**Figure 7:** Eca-109 cell apoptosis amongst control, NC, and siTCF-3 groups (**A**) Cell apoptosis by FCM; (**B**) apoptosis rates of cells; (**C**) gray value of cleaved-caspase-3, Bcl-2, and Bax protein bands; (**D**) protein levels of cleaved-caspase-3, Bcl-2, and Bax; **, *P*<0.01 compared with the control group.

## Discussion

EC is one of the top ten most life threatening and fatal cancers worldwide in which China has the highest occurrence and mortality rate [20]. Despite the traditional therapies, various factors have been detected for their roles in EC such as miRNAs [21] and B7-H1 [22]. And TCF-3 has been discovered as a tumor promoter in several cancers such as colorectal cancer [23] and prostate cancer [24]. Our study investigated the role of TCF-3 in Eca-109 cells, and the results indicated that *TCF-3* gene silencing could significantly inhibit the proliferation and further growth of Eca-109 cells and induces cell apoptosis.

After TCF-3 was silenced by RNAi, the amount of mRNA and protein expression of *TCF-3* gene in Eca-109 cells reduced. RNAi is a remarkably potent method for decreasing endogenously expressed protein, which is widely served for biological applications and for silencing mRNAs encoding pathogenic proteins [25]. As reflected by another study, it was found that after silencing by RNAi, the mRNA and protein expressions of galectin-3 were decreased [12]. And the morphology of Eca-109 cells became irregular with cell membrane crinkled and broken, cells vanished and the cell density also decreased. In general, activating TCF-3 serves as a gene aggravating inflammation [26]. This result indicates that silencing *TCF-3* gene could decrease the number of cancer cells.

Moreover, our study showed that *TCF-3* gene silencing induced arrest of Eca-109 cells in G_0_/G_1_ cell phase and decreased the proliferation of Eca-109 cells. Patel et al. [27] had suggested that silencing of TCF-3 contributed to the decrease in the proliferation of prostate cancer cells, and interestingly, the number of cells in the G_1_-phase significantly increased, whereas the cells in G_2_-phase decreased, which demonstrated the cell cycle arrest of cancer cells was induced and the proliferation was regressed. In EC cells, Wnt1 induced TCF-dependent/β-catenin transcription, and regulated β-catenin expression in EC tissues was found [28]. Abnormal expressions of Wnt signaling pathway components are reported in several cancers, including EC, and it is also involved in cancer development and progression [29]. Furthermore, it has also been proved that β-catenin plays a significant role in the apoptosis of EC cells [30]. Wnt/β-catenin signaling is involved in the activation of target genes by an interaction of β-catenin with TCF-3, and the Wnt pathway plays a major role in controlling cell proliferation [31]. The ability of colony formation of cells decreased in Eca-109 cells after *TCF-3* gene was silenced. It was found that many transcription factors regulated by β-catenin were capable of enhancing the ability of colony formation of cancer cells [32]. Kunmar, S et al. have identified that the high levels of *TCF-3* gene are strongly correlated with basal-like tumors and *TCF-3* gene silencing decreased the ability of cancer cells for initiation of tumor formation, and contributed to reduced rates of tumor growth [14]. TCF-3 silencing relatively slowed down the further growth of gastric cancer cells, and the proliferation rate and colony formation of cells were reduced as well [33].

The apoptosis rate of Eca-109 cells was improved after TCF-3 was silenced, and the expression of apoptosis-related protein Bcl-2 decreased, while caspase-3 and Bax expressions increased. Studies have revealed that the down-regulation of TCF-3 induced cell apoptosis, inhibited cell viability and migration of several tumor cells [34,35]. It has been proved that activating TCF-3 was capable of repressing Bax transcription [36]. Several studies have shown that the increased expression of Bax and caspase would result in cell apoptosis [37,38]. Hossain et al. had identified that the repressed TCF could reduce Bcl_xL_ expression and Bcl-2 could rescue cell apoptosis [39]. And it is also suggested that the high expression of Bcl-2 could relatively prevent cell apoptosis and result in blocking apoptosis induced by various agents in different kinds of cells [40,41].

To sum up, our study proved that as a member of transcription factor family, TCF-3 acts as an advocator and promoter for EC, and the silenced TCF-3 could decrease the growth, viability, colony formation, and proliferation of Eca-109 cells. Besides, the apoptosis rate of Eca-109 cells was enhanced after *TCF-3* gene was silenced. Therefore, silencing *TCF-3* gene might serve as a novel target for EC. However, other factors correlated with TCF-3 and EC were not involved, and also the potential mechanism of *TCF-3* gene silencing in EC is not known yet. Hence, in the future, more studies in this field are needed to identify the mechanism and develop new targets for the treatment of EC.

## Abbreviations

CST: Cell Signaling Technology
BrDU 5: bromo-2-deoxyuridine
EC: esophageal cancer
EP: Eppendorf
FCM: flow cytometry
HRP: horseradish peroxidase
NC: negative control
PBST: PBS containing Tween
PI: propidium iodide
RT-qPCR: reverse-transcription quantitative PCR
siTCF-3: siRNA against TCF-3
TBST: TBS with Tween 20
TCF-3: transcription factor 3
